# The Study on the Pathogenesis of Pediatric Lymphoma Based on the Combination of Pseudotargeted and Targeted Metabolomics

**DOI:** 10.1155/2021/9984357

**Published:** 2021-05-25

**Authors:** Hongqi Sun, Nan Chen, Xuchen Wang, Na Li, Shanshan Wang, Zhengyan Zhang, Ying Zhou, Junmei Yang

**Affiliations:** Zhengzhou Key Laboratory of Children's Infection and Immunity, Children's Hospital Affiliated to Zhengzhou University, Zhengzhou 450018, China

## Abstract

Pediatric lymphoma is a kind of malignant tumor with high mortality. The complexity of pediatric lymphoma shows a great challenge for effective diagnosis and treatment. In order to meet the challenge, the combination of pseudotargeted and targeted metabolomics was used to analyze the serum metabolites in pediatric lymphoma patients and healthy controls for discovering the metabolites related to pediatric lymphoma. The serum samples were obtained from the treatment group (*n* = 43), the control group (*n* = 26), and the patients group (*n* = 18). A total of 17 serum metabolites, including carnitine, leucine, creatine, urea, (6Z,9Z,12Z)-octadecatrienoic acid, linoleate, octadecenoic acid, L-palmitoylcarnitine, hexadecanoic acid, tetradecanoic acid, (9Z)-hexadecenoic acid, uric acid, glucose, 1-methylnicotinamide, hypoxanthine, L-glutamine, and taurine, were found to be related to pediatric lymphoma. They could provide a scientific diagnostic basis and therapeutic target for pediatric lymphoma and elucidate the mechanism of pediatric lymphoma.

## 1. Introduction

Lymphoma is one of the most common pediatric cancers, accounting for nearly one third of all pediatric cancers. It is one of the main causes of death in children ages 1 to 10 [1]. The actual incidence of pediatric lymphoma may be underestimated because of different diagnostic criteria [2]. Lymphoma may be caused by genetic, infectious, and inflammatory etiologies [3]. In 2015, the “second child policy” was adopted in China. The number of children has increased during the past years. The number of pediatric lymphoma patients will significantly increase. However, the pathogenesis of pediatric lymphoma is complex and still unclear. Therefore, it is very necessary to explore the etiology of pediatric lymphoma. The metabolites in serum could be the best representation of the system phenotype [4]. Thorough metabolomics based on mass spectrometry is a powerful tool for diagnosis in cancer disease [5]. To date, there are no available serum metabolomics studies on pediatric lymphoma. There are a large number of metabolites with structural diversity in serum [6]. Therefore, an analytical method with high coverage, high sensitivity, high specificity, and wide dynamic range needs to be developed. Pseudotargeted metabolomics (SWATHtoMRM) using the variable sequential window acquisition of all theoretical fragment-ion spectra (vSWATH) and multiple reaction monitor (MRM) meets the need of high sensitivity, high coverage, good reproducibility, and wide dynamic range [7–9]. In our study, we utilized a combination of pseudotargeted and targeted metabolomics to analyze the serum metabolites in pediatric lymphoma patients and healthy control subjects. Two batches of serum were collected from pediatric lymphoma patients and healthy subjects. One batch of serum was used for pseudotargeted metabolomics analysis. The other batch of serum was used for targeted analysis to validate the biomarkers. At present, little is known about the metabolomics of pediatric lymphoma. Our purpose is to discover potential biomarkers of pediatric lymphoma and give a new perspective to understand the mechanism of pediatric lymphoma. The results may provide valuable information for the diagnosis and personalized treatment of pediatric lymphoma.

## 2. Materials and Methods

### 2.1. Subjects

A total sample size of 87 subjects was estimated by the MetSizeR approach for sample size estimation using the following assumptions: a target false detection rate of 5%, spectra of 1709 spectral bins, and an expected proportion of significant spectral bins of 20% [10]. Subjects (*n* = 87) were recruited from the Children's Hospital Affiliated to Zhengzhou University, from Jan 2020 to June 2020. Children aged 1 to 10 were selected in the study. The subjects were classified as the patients' group (*n* = 18), the treatment group (*n* = 43), and the control group (*n* = 26). The information of the subjects is shown in Table 1. There is no significant difference in gender and age among the three groups. Pediatric lymphoma was diagnosed referring to the 2016 revision to the World Health Organization classification of myeloid neoplasms and acute leukemia [11–13]. Patients were treated with the Chinese Children Cancer Group-non-Hodgkin Lymphoma 2010 protocol. The study was approved by the Ethics Committees of Children's Hospital Affiliated to Zhengzhou University (2021-K-026). The informed consent have been signed by all subjects in the study. Serum samples were acquired and stored at -80°C.

### 2.2. Sample Preparation

In our study, 100 *μ*L of serum samples were mixed with 300 *μ*L of methanol containing internal standards: 100 ng/mL of clenbuterol and chloramphenicol. Then, the mixture was vortexed for 10 min and centrifuged at 14000 × g for 20 min, at 4°C. The supernatant was used for metabolomics analysis.

### 2.3. Pseudotargeted Metabolomics Analysis

In our study, 10 *μ*L of each sample supernatant was mixed and prepared for quality control (QC) samples. Quality control of samples was performed by an ExionLC AD liquid chromatography system coupled with a TripleTOF 5600 system. A Waters UPLC® BEH C_18_ column (2.1 × 100 mm, 1.7 *μ*m) and a Waters UPLC® BEH HILIC column (2.1 × 100 mm, 1.7 *μ*m) were used for LC separation in metabolomics analysis. The total liquid flow rate was set at 0.4 mL/min. The chromatography column temperature was set at 40°C. When the C_18_ column was used for sample separation, mobile phase A consisted of 10 mM ammonium acetate and water containing 0.1% formic acid. Acetonitrile was used as mobile phase B. Then, the elution gradient was as follows: 10% B (0–0.5 min), 95% B (0.5–8.5 min), and 10% B (10–10.1 min). The total elution time was 14 min. When the HILIC column was used for sample separation, mobile phase A consisted of water with 5 mM ammonium acetate. Mobile phase B consisted of acetonitrile. The elution gradient was as follows: 40% A (0–0.5 min), 90% A (0.5–8.5 min), and then 40% A (10–10.1 min). The total elution time was 13 min. Variable SWATH data were obtained from QC samples based on TripleTOF 5600+ mass spectrometry. Then, the SWATH data were converted to MRM transition data files. Then, MRM transitions were performed on a QTRAP 5500 for all serum samples. QC samples were also acquired once every five serum samples. The nebulizer gas was set to 60 psi. The ion spray voltage was set to 5,500 V (in positive mode) and -4500 V (in negative mode). The nebulization temperature was set to 500°C. The DP value was set to 60 V (in positive mode) and -60 V (in negative mode). The CE value was set to 35 ± 15 V (in positive mode) and −35 ± 15 V (in negative mode). The full scanning range was from *m*/*z* 50 to *m*/*z* 1000.

### 2.4. Targeted Analysis

Targeted analysis was also performed by an ExionLC AD system coupled with a QTRAP 5500 system. The LC separation was the same as the pseudotargeted metabolomics. MRM scan mode was used for potential biomarker detections. The MRM transitions and their collision energy are seen in Table 2. The source temperature was set to 500°C. The nebulizer gas was set to 60 psi.

### 2.5. Data Processing and Statistical Analysis

In total, 87 serum samples were analyzed in replicates. The peak area of each feature was acquired using MultiQuant 3.0.3. The source contamination or the maintenance of the mass-spectrometer may affect the analytical reproducibility. Therefore, it is necessary to decrease systematic change using normalization of peak areas of all features. The features (RSD < 15%) in QC samples were selected for statistical analysis. In our study, partial least-squares discriminant analysis (PLS-DA) was used to model all features in MetaboAnalyst (http://www.metaboanalyst.ca). Internal validation with 7-fold cross-validation and response permutation testing were used to test the predictability of the model. Variable importance in the projection (VIP) value of all features was calculated from the best-fitted PLS-DA model. The variables with VIP > 1 and FDR < 0.05 were selected. Student's *t*-test was used for univariate statistical analysis. Variables with univariate statistical significance (*p* < 0.05) were considered as differential variables. The potential differential variables were validated by VIP value and FDR value and *p* value. These variables were identified according to their accurate mass, isotope ratio, and fragmentation ions. The databases including KEGG, PubChem compound, METLIN, the Madison Metabolomics Consortium Database, and the Human Database were used to search them [14].

In our study, targeted metabolomics data were extracted by MultiQuant 3.0.3. The internal standards were used to calibrate the concentrations of potential biomarkers. Multivariate statistical analysis was also performed with MetaboAnalyst. PLS-DA was applied to distinguish the pediatric lymphoma patients' group and the treatment group. The differences of biomarkers (VIP > 1 and *p* < 0.05) were considered to be significant between the two groups. The relationship between the different biomarkers were illustrated with the MetaboAnalyst software [15].

## 3. Results

### 3.1. Analytical Characteristics of Pseudotargeted Metabolomics Method

Internal standards were used to assess the reliability of the pseudotargeted metabolomics method. Internal standards were added to the serum sample. The linear curves of internal standards were calculated by their peak area at each concentration. The results displayed that the linear regression coefficients of internal standards were all more than 0.99. The linear relationship was very good. The recovery of the analytical method was assessed using low, medium, and high concentrations of internal standards in six replicates. Our results displayed that the recoveries ranged from 87.6% to 112.7% for internal standards at each concentration. The recovery of our pseudotargeted metabolomics method was very good. The relative standard deviation (RSD) of peak areas of QC samples was used to evaluate the repeatability of the analytical method. In our study, all features occurred at RSD < 14%. Therefore, our pseudotargeted metabolomics method was suitable for pediatric lymphoma serum detection.

### 3.2. Children Serum Pseudotargeted Metabolomics

For pseudotargeted metabolomics, serum was analyzed by UPLC-TripleTOF 5600+ and QTRAP 5500. The typical total ion chromatographs of serum samples are shown in Figure 1, indicating that the chromatography separation was excellent. The corresponding SWATH data of the metabolites were used to identify them based on their accurate mass, isotope ratio, and fragment-ion spectra. For example, M1 displayed the [M − H]^−^ ion at *m*/*z* 124.0080. Its elution time was 4.7 min. The molecular formula of M1 was inferred as C_2_H_7_NO_3_S based on its accurate mass and isotope ratio. A series of product ions were observed at *m*/*z* 106.9802, 79.9578, and 64.9699, as seen in Figure 2. The fit of fragment-ion matching was greater than 85%. The structure of M1 could be inferred as taurine. QC samples were inserted in every ten samples for evaluating the reproducibility of the analytical platform. As seen in Figure 3, QC samples were tightly located in the score plot of the PLS-DA mode, indicating that the reproducibility of our analytical method was very good. As seen in Figure 3, the patients' group was well separated from the treatment group and healthy control group on the PC1 dimension. It indicates that some features in the patients' group have been changed. The score plot and loading plot of PLS-DA analysis between the patients' group and the treatment group are shown in Figures 4 and 5. The VIP scores of each metabolite are shown in Figure 6. The 17 features (VIP value > 1 and *p* value < 0.05) were selected as the potential differential metabolites. The heat map is also shown in Figure 7. The 17 differential features were identified as carnitine, leucine, creatine, urea, (6Z,9Z,12Z)-octadecatrienoic acid, linoleate, octadecenoic acid, L-palmitoylcarnitine, hexadecanoic acid, tetradecanoic acid, (9Z)-hexadecenoic acid, uric acid, glucose, 1-methylnicotinamide, hypoxanthine, L-glutamine, and taurine. Their retention times and fragment ions were confirmed using the standard compounds from Sigma-Aldrich.

### 3.3. Children Serum Targeted Metabolomics

The 17 potential metabolites in serum were measured using QTRAP 5500. Their differences between the treatment group and the patients' group were validated through statistical analysis. These 17 potential differential metabolites were verified to be significantly different in content between the treatment group and the patients' group. In the patients' group, 14 metabolites, namely, carnitine, leucine, creatine, urea, (6Z,9Z,12Z)-octadecatrienoic acid, linoleate, octadecenoic acid, L-palmitoylcarnitine, hexadecanoic acid, tetradecanoic acid, (9Z)-hexadecenoic acid, uric acid, 1-methylnicotinamide, and hypoxanthine were upregulated, and 3 metabolites, namely, L-glutamine, taurine, and glucose, were downregulated. The differences in the 17 metabolites between the treatment group and the patients' group are shown in Figure 8 with GraphPad Prism [16]. The relationship of the 17 potential metabolites with pediatric lymphoma will be described in the following discussion.

### 3.4. Metabolic Pathway Analysis

MetaboAnalyst was used for metabolic pathway analysis. In our study, an abnormal metabolic pathway was involved in fatty acid metabolism, fatty acid biosynthesis, mitochondrial beta-oxidation of long-chain saturated fatty acids, purine metabolism, and taurine and hypotaurine metabolism, as seen in Figure 9. The AUC value in validation data was more than 0.8, with a sensitivity of 85%. Metabolic pathways were intensively studied to gain insight into the disturbed metabolism of pediatric lymphoma.

## 4. Discussion

Traditional untargeted metabolomics and targeted metabolomics were often explored to detect as many metabolites as possible and accurately quantify known metabolites, respectively. However, the untargeted metabolomics method had encountered great challenges in the detection of metabolites in a wide range of concentrations [17]. The limitation of targeted metabolomics is primarily low coverage [18]. Therefore, in our study, the pseudotargeted metabolomics (SWATHtoMRM) method with good reproducibility, high sensitivity, high coverage, and a wide dynamic range was explored to detect the metabolites in serum. Targeted metabolomics was used to validate the results of pseudotargeted metabolomics. Pseudotargeted metabolomics and targeted metabolomics were applied to discover new biomarkers and investigate the pathogenesis for pediatric lymphoma diagnosis and prognosis.

The etiology and diagnosis of pediatric lymphoma is complex [19]. Yang et al. displayed that metabolites associated with amino acid metabolism, energy metabolism, choline phospholipid metabolism, and fatty acid metabolism were altered in Burkitt lymphoma mice [20]. Glutamate, glycerol, choline, pyruvate, lysine, creatine, *α*-ketoglutarate, betaine, glycine, lactate, serine, tyrosine, glucose, phenylalanine, histidine, leucine, and isoleucine were the potential diagnostic biomarkers using analyzing serum untargeted metabolomics of Burkitt lymphoma mice models. Stenson et al. used serum ^1^H nuclear magnetic resonance metabolomics to find that lysine, arginine, 2-hydroxybutyrate, aspartate, valine, ornithine, and pyroglutamate are altered in diffuse large B-cell lymphoma patients [21]. However, little literature about pseudotargeted metabolomics of pediatric lymphoma were reported.

In our study, the PLS-DA score plot showed that the levels of leucine and creatine are higher in pediatric lymphoma patients than in the treatment group, and the content of glucose becomes lower in pediatric lymphoma subjects than in the treatment group. The content of leucine was increased due to the interaction among different amino acid pools in the tumor [20]. Leucine belongs to branched chain amino acids. It was used for the anaplerosis in the tricarboxylic acid cycle in tumor growth. The deficiency of leucine will hamper the proliferation of tumor cells. In order to meet the requirements for tumor cell growth, creatine could provide substrates for energy synthesis [22]. Moreover, the content of creatine and glucose was increased in pediatric lymphoma patients in our study. Glucose is metabolized to pyruvate by glycolysis. However, pyruvate does not enter the tricarboxylic acid cycle. It is transformed to lactate or alanine. Aerobic glycolysis is increased in tumor cells [23].

Fatty acids are important sources of fuel to produce adenosine triphosphate in mitochondria using carnitine as a medium [24]. In our study, the level of carnitine, L-palmitoylcarnitine, (6Z,9Z,12Z)-octadecatrienoic acid, octadecenoic acid, hexadecenoic acid, tetradecanoic acid, and (9Z)-hexadecenoic acid are all higher in pediatric lymphoma patients than in the treatment group. They belong to the fatty acid metabolism, fatty acid biosynthesis, and mitochondrial beta-oxidation of the long-chain saturated fatty acid pathway. According to our results, abnormal fatty acid metabolism occurs in tumor cells. A previous study has displayed that high levels of fatty acid synthase and endogenous fatty acid synthesis were expressed in cancer cells [25]. Bioenergy can be delivered by the oxidation of the fatty acids for tumor cell proliferation [25, 26]. It indicated that mitochondrial dysfunction was associated with pediatric lymphoma.

In addition, we found that the levels of urea, uric acid, and hypoxanthine are higher in pediatric lymphoma patients than in the treatment group, and the content of L-glutamine becomes lower in pediatric lymphoma patients than in the treatment group. They belong to the purine metabolism pathway. Uric acid is increased in pediatric lymphoma patients because of the increased turnover of cells, which is consistent with a previous study [27]. The level of taurine is lower in pediatric patients than in the treatment group. Taurine is a potent antioxidant. The significance of taurine and hypotaurine metabolism suggests oxidative stress following treatment [28]. The level of 1-methylnicotinamide is higher in pediatric lymphoma patients than in the treatment group. However, its relationship with pediatric lymphoma is still unclear.

In our study, the pseudotargeted metabolomics based on the advanced SWATHtoMRM method could provide high coverage and high sensitivity for exploring the potential differential metabolites between the pediatric lymphoma patients and the healthy controls. Carnitine, leucine, creatine, urea, (6Z,9Z,12Z)-octadecatrienoic acid, linoleate, octadecenoic acid, L-palmitoylcarnitine, hexadecanoic acid, tetradecanoic acid, (9Z)-hexadecenoic acid, uric acid, glucose, 1-methylnicotinamide, hypoxanthine, L-glutamine, and taurine were identified. However, one limitation may be considered in our study. The number of subjects was relatively small. In further studies, a larger amount of subjects with pediatric lymphoma should be recruited to verify our results. Thus, the present study could only provide indirect evidence for the mechanism of pediatric lymphoma.

## 5. Conclusion

Our study displays that serum metabolomics can play an important role in differentiating patients with pediatric lymphoma from healthy controls. It indicates that the differential serum metabolites may be novel and important biomarkers of pediatric lymphoma to identify pediatric lymphoma. The 17 differential metabolites associated with pediatric lymphoma may provide an improved understanding of the pathogenesis of pediatric lymphoma.

## Figures and Tables

**Figure 1:** The typical total ion chromatographs of serum samples.

**Figure 2:** The comparison of the experimental MS/MS spectrum with the standard MS/MS spectrum of taurine.

**Figure 3:** The score plot of PLS-DA among the healthy control group, the patients' group, and the treatment group.

**Figure 4:** The score plot of PLS-DA between the patients' group and the treatment group.

**Figure 5:** The loading plot of PLS-DA between the patients' group and the treatment group.

**Figure 6:** The VIP score of each biomarker to the discrimination between the patients' group and the treatment group.

**Figure 7:** The hierarchical clustering heat map of the biomarkers.

**Figure 8:** The box plot of 17 metabolites between the patients' group and the treatment group.

**Figure 9:** The metabolic pathways related to pediatric lymphoma.

**Table 1:** The information of subjects.

Groups	Age (years)	Gender
Healthy controls (*n* = 26)	5.7 ± 2.3	19 boys, 7 girls
Patients' group (*n* = 18)	5.5 ± 2.9	13 boys, 5 girls
Treatment group (*n* = 35)	5.9 ± 2.4	27 boys, 8 girls

**Table 2:** MRM transitions, collision energy, and precision of the method.

Compounds	*T*_*R*_ (min)	Parent ion	Product ion	CE (eV)	Precision RSD%
Taurine	4.7	124.0	80.0	-34	7.4%
Leucine	5.8	130.1	112.0	33	8.0%
Creatine	6.2	132.0	90.0	30	5.0%
Urea	0.66	61.1	44.2	40	4.7%
(6Z,9Z,12Z)-Octadecatrienoic acid	9.2	279.2	95.0	-26	7.7%
Linoleate	1.4	281.0	81.0	39	12.6%
Octadecenoic acid	10.0	283.3	69.0	37	9.2%
L-Palmitoylcarnitine	8.0	400.3	85.0	42	4.6%
Hexadecanoic acid	9.7	257.2	57.0	34	12.0%
Tetradecanoic acid	1.5	229.1	211.2	17	4.5%
(9Z)-Hexadecenoic acid	1.4	255.1	237.1	20	5.0%
Uric acid	4.4	167.0	124.0	-22	6.5%
Glucose	3.2	179.1	89.1	-36	3.3%
1-Methylnicotinamide	3.0	137.1	94.0	32	11.5%
Hypoxanthine	1.1	137.0	110.0	21	12.0%
L-Glutamine	6.7	145.1	127.0	-19	9.5%
Carnitine	6.9	162.1	103.0	26	8.5%

## Data Availability

The datasets in our study are available from the corresponding author on reasonable request.
